# Facile Fabrication of CuO Nanoparticles Embedded in N-Doped Carbon Nanostructure for Electrochemical Sensing of Dopamine

**DOI:** 10.1155/2022/6482133

**Published:** 2022-10-14

**Authors:** Nebras Sobahi, Mohd Imran, Mohammad Ehtisham Khan, Akbar Mohammad, Md. Mottahir Alam, Taeho Yoon, Ibrahim M. Mehedi, Mohammad A. Hussain, Mohammed J. Abdulaal, Ahmad A. Jiman

**Affiliations:** ^1^Department of Electrical & Computer Engineering, Faculty of Engineering, King Abdulaziz University, Jeddah 21589, Saudi Arabia; ^2^Department of Chemical Engineering, College of Engineering, Jazan University, P.O. Box 706, Jazan 45142, Saudi Arabia; ^3^Department of Chemical Engineering Technology, College of Applied Industrial Technology (CAIT), Jazan University, Jazan 45971, Saudi Arabia; ^4^School of Chemical Engineering, Yeungnam University, Gyeongsan-si, Gyeongbuk 38541, Republic of Korea; ^5^Center of Excellence in Intelligent Engineering Systems (CEIES), King Abdulaziz University, Jeddah, Saudi Arabia

## Abstract

In the present study, a highly selective and sensitive electrochemical sensing platform for the detection of dopamine was developed with CuO nanoparticles embedded in N-doped carbon nanostructure (CuO@NDC). The successfully fabricated nanostructures were characterized by standard instrumentation techniques. The fabricated CuO@NDC nanostructures were used for the development of dopamine electrochemical sensor. The reaction mechanism of a dopamine on the electrode surface is a three-electron three-proton process. The proposed sensor's performance was shown to be superior to several recently reported investigations. Under optimized conditions, the linear equation for detecting dopamine by differential pulse voltammetry is *I*_pa_ (*μ*A) = 0.07701 *c* (*μ*M) − 0.1232 (*R*^2^ = 0.996), and the linear range is 5-75 *μ*M. The limit of detection (LOD) and sensitivity were calculated as 0.868 *μ*M and 421.1 *μ*A/*μ*M, respectively. The sensor has simple preparation, low cost, high sensitivity, good stability, and good reproducibility.

## 1. Introduction

Dopamine (DA) is a common hormone in the family of catechol ethylamine which works as a neurotransmitter. It affects the renal, nervous, and cardiovascular systems as well as endocrine system of mammals [1]. DA controls certain physiological conditions, *such as* movement, learning, memory, behavior, mood, and mental cognition [2, 3]. DA excites the heart and increases the blood flow. When dopamine (DA) levels are low, people lose the ability to control muscles and continue to tremble. In severe cases, this leads to Parkinson's, Alzheimer's, schizophrenia, and other symptoms [2, 4]. The neurological disorders, depression, autism, congenital cardiopathy, hypertension, bronchial asthma, and septic shock are treated using DA clinically [5]. Due to such important uses and function of DA in human body, it is necessary to detect DA concentration very accurately. Among various methods of detection, electrochemical sensing is a proficient method which detects the biological molecules in very low detection range with high sensitivity and good selectivity [6, 7]. Nanoparticles play an important role in electrochemical detection and are widely used in electrode fabrication for chemical sensors and bio-sensors [8–11]. Apart from electrochemical sensing applications, nanostructured materials are extensively used in various applications, *such as* heat transfer, photocatalysis, hydrogen production, solar cell, biomedical equipment, and therapeutics [12–20]. Various electro catalysts have performed efficiently in electrochemical-based sensors and contributing in this technique since decades [21, 22].

In the catalytic analysis of small biological molecules, the sensitivity is improved to a certain extent and the detection limit is lowered. However, the expensive precious metal price limits the further popularization of these research results. Reducing costs and getting to the goal quickly and efficiently without reducing catalytic performance is one of the current problems facing by analysts. Compared to noble metals (*such as* Pt and Au), Cu is preferred because of its advantages *such as* great elasticity, good toughness, high wear resistance, affordable price, and good electrical conductivity. On this basis, CuO nanoparticles were embedded into the nitrogen-doped carbon matrix, and as a new nanocomposite material CuO@NDC was synthesized. Previous research found that adsorption of pollutants over the surface of the catalysts promotes the effectiveness. The doped-carbon materials can help for the surface adsorption and enhance the charge transfer process. In addition to this, nitrogen-doped carbon materials can participate in higher conductivity and improve electron transport, resulting in a potential electrode material for electrochemical sensing applications [23, 24]. As a consequence, the produced CuO@NDC nanocomposite, which combines the benefits of high conductivity N-doped carbon and unusual properties of CuO, may significantly improve electrochemical sensing performance [24].

When CuO nanoparticles are dispersed into N-doped carbon matrix, they show higher catalytic activity due to the synergy between the two. This material is used to modify the glassy carbon electrode and the DA content using differential pulse voltammetry.

## 2. Experiment

### 2.1. Reagents

Copper nitrate trihydrate (Cu(NO_3_)_2_.3H_2_O) (99.5%), concentrated sulfuric acid (H_2_SO_4_) (98.5%), and sodium hydroxide (NaOH) (99%) were purchased from Sigma Aldrich, USA. The other reagents *such as* dopamine (DA) (99.5%), ascorbic acid (AA) (99%), uric acid (UA) (99.5%), sodium chloride (NaCl) (98.5%), urea, and glutaraldehyde were purchased from Sinopharm Chemical Reagent Co Ltd, China.

### 2.2. Preparation of NDC and CuO@NDC

The method was used to fabricate the samples with certain modifications as reported in the literature [23, 25]. The polymeric metal complex was used to fabricate the nanocomposite. 1.20 g urea and 4.00 mL glutaraldehyde in a basic medium (at pH 8-9) were used to make the polymer-metal complex. 1.87 g copper(II) nitrate was added to the polymer matrix and heated at 60°C for 6 hours to get the polymer copper(II) complex. The hydrothermal method was adopted to fabricate the hydrochar, a 100 ml autoclave was filled with 3.00 gm of polymer Cu (II) complex, and 20 ml of distilled water was added and sealed properly, and the autoclave was heated to 250°C for 24 hours. After that, the autoclave was cooled and the resulting hydrochar was filtered, washed, and dried before being used for further heat treatment to produce the graphite carbon matrix. The resultant hydrochar was heated to 800°C at a rate of 5°C/min under argon flow and held at that temperature for 1 hour. Before use, the CuO@NDC was vacuum dried for 24 hours. NDC was produced without Cu(II) source using a similar method [23, 25].

### 2.3. Characterization

The powder X-ray diffraction (XRD) pattern of the as-synthesized nanocomposites powder was recorded using a Rigaku Ultima IV diffractometer (Cu K radiation). The FT-IR spectra were recorded in transmission mode on a Bruker Tensor spectrometer using KBr pellets with a scan range of 400-4000 cm^−1^. Raman spectra were recorded on Aramis LabRam spectrometer. The Brunauer-Emmett-Teller (BET) technique of N_2_ adsorption isotherms at 77.35 K; the Quantachrome Autosorb-1-MP analyzer was utilized to measure the aperture characteristics and specific surface area of the nanocomposite. Field emission scanning electron microscopy was used to study the shape and structure of manufactured materials (FESEM, JEOL, JSM-7600F). The samples were imaged and studied using a transmission electron microscope (TEM/HRTEM, JEOL, JEM-2100F) operating at 120 kV. The X-ray photoelectron spectroscopy (XPS) experiment was carried out with the help of ESCALAB250 equipment outfitted with an Al K X-ray source.

### 2.4. Fabrication of CuO@NDC Electrode

The cyclic voltammetric (CV), differential pulse voltammetry (DPV), and electrochemical impedance spectroscopy (EIS) were carried out at room temperature utilizing a CHI660C electrochemical workstation equipped with a three-electrode setup. The glassy carbon electrode (GCE) having 3 mm diameter was prepared by polishing alumina slurry and washed off with ethanol and distilled water and dried at room temperature. Thereafter, 10 *μ*L of the nanocomposite suspension made using ethanol Nafion solution (0.5 mg/mL) was drop cast over the surface of GCE and dried at room temperature.

The cyclic voltammetry analysis was performed at several scanning rates ranging from 10 to 200 mV/s between 0.0 and + 0.8 V using 0.1 M NaOH solution as the background electrolyte. Individual CV tests were performed by adding 0.1 mL of newly produced aqueous solution of the DA analyte to 10 mL of 0.1 M NaOH medium. EIS measurements were carried out in solution of 5 mmol/L [Fe(CN) 6]^4−^/[Fe(CN) 6]^3−^ in 0.1 mol/L KCl at a bias potential of 0.55 V using an AC voltage with a 5 mV amplitude in the frequency range of 0.1 Hz to 1 MHz. At low concentrations, interfering species *such as* ascorbic acid, glucose, uric acid, glutamic acid, and sodium chloride were also investigated.

## 3. Results and Discussion

Figure 1(a) shows the XRD pattern of NDC and Cuo@NDC. The diffraction peak at 25.6 degree of two theta is assigned to the (002) crystallographic plane of graphite. The CuO@NDC prepared by hydrothermal method shows the diffraction peaks at the value of two theta which are 35.5, 38.6, 48.7, 53.2, 58.1, 61.3, 66.1, 68, 72.2, and 75.0 corresponding to the (−111), (111), (−202), (020), (202), (−113), (−311), (220), (311), and (−222) crystallographic planes, respectively (JCPDS, No. 41-0254) [26]. These featured peaks obtained at the specified two theta values suggest the successful formation of CuO@NDC nanostructures. The crystal size calculated using Scherrer's equation was obtained ∼21.5 nm for the highest peaks observed. The FTIR spectra of NDC and CuO@NDC are shown in Figure 1(b). The bands appeared at 626 cm^−1^ and 434 cm^−1^ ascribed to the vibration of Cu-O functional group [27]. The stretching vibrations of O-H functional group suggested at the ∼3400 cm^−1^ which is appeared as a broad band in the spectrum of both NDC and CuO@NDC. The strong band that appeared at 1625 cm^−1^ is due to the overlapping of bending vibrations of N-H and stretching vibrations of C = O in amide band [27]. The band that appeared in NDC at 1594 cm^−1^ is disappeared or shifted to 1625 cm^−1^ in nanocomposite due to heat treatment decompose-NHCO group [27]. The bands that appeared at 1424 cm^−1^ and 1147 cm^−1^ suggest the deformation vibration of C = N and C-N bonds, respectively, which indicate the successful synthesis of nitrogen doping in the carbon matrix [27]. The slight shifting of bands in the CuO@NDC nanocomposite confirms the successful decoration of CuO in NDC.

To evaluate the structure of the nanocomposites, the effective measurement of nanocomposite was employed in the form of Raman spectroscopy and the results are presented in Figure 1(c). Two intense peaks were observed, which are attributed to *D* and *G* bands, respectively. The *D* band appeared at 1350 cm^−1^ and *G* band appeared at 1594 cm^−1^ corresponding to the sp^2^-bonded carbon atoms which indicate a disordered graphitic structure and sp^3^ carbon atom, respectively [28]. There are total 3 modes (*Ag*^+2^*Bg*) that are Raman active in CuO nanoparticles [29–32]. The other strong peak observed at 284 cm^−1^ is *A*_1_*g* Raman active optical-phonon *Ag* mode of monoclinic (C_2_/c) CuO NPs. The other significant peaks were observed at 332 cm^−1^ and 614 cm^−1^ which are known as *B*_1_*g* and *B*_2_*g* modes, respectively [33]. The porosity, surface area, and other properties of CuO@NDC nanocomposite were obtained by N_2_ sorption isotherm at 77 K as presented in Figure 1(d). The isotherm of the characterized sample was found to be following the mesoporous sample. Brunauer–Emmett–Teller surface area was calculated for the nanocomposite and was obtained SBET = 140.32 m^2^/g. The high surface area can be attributed to the dense network of the CuO-decorated NDC matrix. Furthermore, the total pore volume of the CuO@NDC NC was found to be 0.424 cm^3^/g. The large surface area, pore volume, and hierarchical pore structure were very beneficial to the exposure of active sites and rapid transportation of gas molecules to catalytic sites [34, 35].

Figure 2(a) represents the SEM image of the CuO@NDC, which states about the morphology and surface topology of the nanocomposite. The image shows that the CuO nanoparticles are embedded in the nitrogen-doped carbon matrix. The network of carbon matrix is so dense, and the CuO nanoparticles are decorated uniformly on the nitrogen-doped carbon nanostructures, which indicate the successful formation of CuO@NDC. The TEM images are shown in Figure 2(b), which shows that the dark images of spherical-shaped CuO nanoparticles are embedded in a nitrogen-doped carbon network. The size of CuO nanoparticles was found to be ∼15 nm. The HRTEM (Figure 2(c)) shows the lattice spacing of CuO, and it was found to be 0.25 nm, which is corresponding to the (002) crystallographic plane of CuO [26].

The XPS analysis is presented in Figure 3 and shows the survey scan, C, N, O, and Cu elements. The peaks for C, N, O, and Cu were obtained at ∼284.8 eV, 400.06 eV, 531.5 eV, and 934.6 eV, respectively, which are presented in Figure 3(a), which indicates the successful decoration of CuO@NDC. Further, deconvolution of the C 1s, N 1s, O 1s, and Cu 2p spectra is carried out to understand the atom-binding states in the CuO@NDC nanocomposite. Four components of C 1s exist in CuO@NDC, corresponding to the graphite-like sp^2^ C--C at 284.7 eV, 285.7 eV, 287.2 eV, and 289.07 eV, which are presented in Figure 3(b). Similarly, Figure 3(c) represents the three components of N 1s which can be found to exist at 399.5, 400.5, and 402.07 that are ascribed-NH_2_/pyridine, pyrrolic N/or graphitic N, and pyridine-N-oxide, respectively [36]. The deconvolution of 2p peaks of Cu can be done into 934.6 eV, for Cu 2p_3/2_ and for Cu 2p_1/2_ at 954.4 eV, while their satellite peaks can be observed at 943.4 eV and 962.4 eV, as shown in Figure 3(d). The high-resolution spectrum of O 1s can be seen in Figure 3(e) where three peaks centered at 529.4 eV, 531.2 eV, and 532.7 eV are assigned to the O 1s spectrum, respectively.

### 3.1. Electrochemical Sensing Performance

The dopamine (DA) sensing performance was carried out at different modified electrodes as shown in Figure 4(a). The cyclic voltammetry (CV) (10 *μ*M of DA) results revealed that in the case of glassy carbon electrode (GCE), the very small redox peaks were observed, while in the case of nanocomposite the intensity of these peaks was increased and the CuO@NDC redox peaks show higher current density. The sensing of the DA was characterized at different scanning rates and was carried out in the range of 25-200 mV/s. It was noticed that as the scanning rate was increased, the current density of the redox peak was increased linearly. The linear equations of redox peak current and sweep rate are *I*_pa_ = 0.00908 *v* + 0.6259 (*R*^2^ = 0.9679) and *I*_pc_ = −0.0176 *v* − 0.8764 (*R*^2^ = 0.9633). The results reveal that the current density of the redox peak increased linearly as the scanning rate was increased [37, 38]. The linear equations of the logarithm of scan rate and redox peak potential were determined using the following Laviron Equation [39] as shown in Figure 4(f).

(1) $$\begin{array}{c} E_{pa}\left(V\right)=0.0296\;\log v\left(Vs^{-1}\right)+0.351\left(R^{2}=0.9916\right), \end{array}$$

(2) $$\begin{array}{c} E_{pc}\left(V\right)=-0.0486\;\log v+0.0657\left(R^{2}=0.9961\right), \end{array}$$

where *E*_pa_ and *E*_pc_ represent the oxidation peak potential and the reduction peak potential, respectively, and *v* is the scan rate, The number of electron transferred coefficient (*n*) was obtained from Equation as below:

(3) $$\begin{array}{c} \ln v=\frac{2.3\text{RT}}{n\alpha F}, \end{array}$$

where *α* is the charge transfer coefficient, *n* is the number of electrons transferred, *T* is the Kelvin temperature (273.16 K), *F* is the Faraday constant (96480 C/mol), and *R* is the molar gas constant (8.314 J/(mol/K)). The slope of the plot of *E*_pa_ against log *v* was used for obtaining the value of *n*. The values of *n* and *α* were obtained as 3.17 and 0.0136, respectively. This value of *n* (∼3) means that three electrons were transferred during the redox process [38].

The differential pulse voltammetry (DPV) was also utilized for the detection of DA at different concentrations, and the DPV response results are illustrated in Figure 4(d). The experimental data on varying concentration of DA was make fitted with linear, represented in Figure 4(e) and natural logarithm of scan rate versus potential has shown in Figure 4(f). The results reveal that as the DA concentration was increased, the current density of the oxidation peak was also increased. It shows a good linear relationship in the range of 5∼75 *μ*M. The linear equation is *I*_pa_ (*μ*A) = 0.07701 *c* (*μ*M) − 0.1232 (*R*^2^ = 0.996), and the detection limit was found to be 0.868 *μ*M.

An interference experiment during the detection of DA (25 *μ*M) was carried out in the presence of glucose, ascorbic acid (AA), glutamic acid, NaCl, and uric acid (UA) (Figure 5(a)). The results revealed that in the presence of glutamic acid (GA), ascorbic acid (AA), and uric acid (UA), no change in peak potential and current density was observed, suggesting that the fabricated electrode, CuO@NDC, has the excellent anti-interference ability and is expected to be used in real sample measurement. Although detection of DA in real sample is still challenging owing to its lower range in body fluids, moreover DA is found with many interfering species *such as* UA, AA, and other analytes. The coexistence of other analytes makes it difficult to detect, and therefore, an accurate, rapid, high sensitivity, and high selectivity sensors need to be developed.

Fayemi et al. [40] have analyzed the electrochemical detection of DA using polyaniline (PANI)-metal oxide (MO)-based nanocomposites (where MO = NiO, ZnO, and Fe_3_O_4_). The best sensitivity and limit of detection were found about 0.153 × 10^−7^ M. Due to the best detection limit, it is suggested that this sensor can be applied for real sample measurement. In another study, Minta et al. [41] have proposed the A ternary polyaniline/Fe_2_O_3_-SnO_2_/reduced graphene oxide (PFSG) sensor for the detection of DA in the presence of other interference. The proposed sensor provides the simultaneous detection of DA and UA and the OD was measured as 0.15 *μ*M and 6.4 *μ*M, respectively. The authors have suggested the possibility of detecting DA in presence of other analytes due to good results. Due to nearby range of detection of DA, the current study also suggest to investigate the real sample analysis with modification in the sensor design and other parameters.

The stability and reproducibility measurement of CuO@NDC nanocomposite during DA detection were measured every 5 days, and the parallel experiments were carried out each time. As shown in Figure 5(b), the results showed that the response remains around ∼96.6% after 25 days. These outcomes showed that the produced nanocomposite has excellent stability due to the synergistic effect between CuO nanoparticles and the N-doped carbon.

## 4. Electrocatalytic Responses Using EIS Analysis

The semicircle diameter at high frequency can be used to calculate the electron-transfer resistance at the electrode surface, whereas the slope of the tail line at low frequency can be used to calculate the semi-infinite diffusion of species to the modified electrode [42]. As shown in Figure 6, the plot of NDC/GCE has a smaller semicircle diameter than CuO-NDC/GCE, indicating that CuO-NDC/GCE has a lower electron transfer resistance. Furthermore, the plot of CuO-NDC/GCE in the low frequency tends to be more vertical to the real axis than CuO-NDC/GCE in the high frequency, indicating a higher ion diffusion rate due to the nitrogen-doped carbon nanostructures with good surface conductivity. An equivalent circuit (inset) was fitted with the EIS data (Figure 6). EIS data was fitted with ZSimpWin 3.20 d program and an equivalent circuit (inset) was drawn (Figure 6). Rct and Cdl represent charge transfer resistance and double-layer capacitance, respectively, and Zw is the vector sum of resistance and capacitive reactance, as shown in the circuitry. The experimental values obtained from the impedance data were combined with the EIS fitting data obtained from the equivalent circuits. When compared to NDC, the Rct fitting values for CuO@NDC nanocomposite decrease. The charge-transfer resistance is significantly reduced by embedding NDC into CuO nanoparticles, as evidenced by the nanocomposite's small Rct value, which is much lower than that of bare NDC. The Cdl values tend to trend in the opposite direction as Rct values [43, 44]. The high electron transfer efficiency is indicated by the low Rct and high Cdl values, which further supports the hypothesis.

## 5. Conclusion

In this study, novel nanocomposites (CuO@NDC) were fabricated using the hydrothermal method and used for the electrochemical detection of DA. The results revealed that the DA concentration has a good linear relationship with its peak current, and the LOD and sensitivity were found to be 0.868 *μ*M (S/N = 3) and 421.1 *μ*A/*μ*M, respectively. Strong anti-interference ability, UA, and AA do not interfere with the measurement for the detection of DA. The electrode stability is found good and checked for the modified electrode after storing for several days and retained up to 98.6% on 10^th^ day and maintained up to 96% even after 25 days.

## Figures and Tables

**Figure 1:** (a). XRD of NDC and CuO@NDC, (b) FTIR spectra of NDC and CuO@NDC, (c) Raman spectra of NDC and CuO@NDC, and (d) N_2_ adsorption and desorption isotherm of NDC and CuO@NDC.

**Figure 2:** (a) SEM of CuO@NDC, (b) TEM of CuO@NDC, and (c) HRTEM of CuO@NDC.

**Figure 3:** XPS spectra of CuO@NDC: (a) Survey scan, (b) C 1s spectra, (c) N 1s spectra, (d) Cu 2p spectra, and (e) O 1s spectra.

**Figure 4:** (a) Cyclic voltammograms of GCE, NDC, and CuO-NDC with DA at 100 mV/s scan rate, (b) cyclic voltammograms of CuO-NDC at different scan rates (25, 50, 75, 100, 125, 150, 175, and 200 mV/s), (c) relationship between redox peak current and scan rate (*v*); (d) differential pulse voltammograms of different concentrations of dopamine on CuO@NC electrode in electrolyte solution, (e) plot of current versus concentration of DA, and (f) relationship between the peak potential (*Ep*) and the natural logarithm of scan rate.

**Figure 5:** (a) Interference study for the detection of DA and (b) stability of the sensor (CuO-NDC/GCE).

**Figure 6:** EIS of NDC/GCE and CuO-NDC/GCE in 0.1 M KCl electrolyte solution containing equimolar 1 mM [Fe(CN)].

## Data Availability

The data used to support the findings of the study are available upon request.
